The article "Analysis of the Government and Capital Market's Response to Normalized Epidemic Prevention and Control Based on the Development of Smart Health Care" was published in 2022. Journal: J Healthc Eng.

# Analysis of the Government and Capital Market's Response to Normalized Epidemic Prevention and Control Based on the Development of Smart Health Care

**DOI:** 10.1155/2022/8122322

**Published:** 2022-11-21

**Authors:** Xinzhi Wang, Xiaoqi Wang, Jian Li, Rui Song

**Affiliations:** ^1^School of Management, Tianjin University of Technology, Tianjin, China; ^2^College of Management and Economics, Tianjin University, Tianjin, China

## Abstract

With the continuous prominence of medical problems, the construction of a smart medical system has received more and more attention. With coronavirus disease 2019 in a state of regular prevention and control, the epidemic prevention and control in China had produced favorable effects. Therefore, a comprehensive evaluation of the emergency governance mechanism in China was crucial to epidemic prevention and control worldwide. This paper empirically analyzed the effects of epidemic prevention and control based on the dual perspective of epidemic governance and capital market, taking the daily outbreak data at the provincial level in China as the sample. The findings were as follows: (1) The accumulation of epidemic medical treatment experience in each province and city produced a positive emergency effect on preventing and controlling the dissemination of epidemic. The effective medical security mechanism was one of the most important mechanisms for the significant emergency effect, with the effective material security as a critical supplement. (2) Companies and corporations with stronger capabilities for emergency medical treatment received more positive responses from the capital market comparatively. Aiming at diversifying directions and measurements for the improvement of emergency governance, this paper provided theoretical bases for improving the emergency governance system against major public health emergencies by using the Chinese characteristics.

## 1. Introduction

Since the coronavirus disease 2019 (COVID-19) was declared as a major global public health emergency in late 2019, the epidemic situation has had a significant impact on the economy and medical systems of the concerned countries. The initial lack of awareness of the danger and speed of transmission led to a widespread outbreak and an alarming rate of transmission of COVID-19 [1]. In response to this major public health emergency, China prudently insisted on the organic combination of normalized precise prevention and control and local emergency treatment and the transformation of prevention and control to normalized prevention and control. It established a normalized prevention and control mechanism for rapid disposal, precise control, and effective treatment [2], thus providing its answer to the world [3].

The article "Analysis of the Government and Capital Market's Response to Normalized Epidemic Prevention and Control Based on the Development of Smart Health Care" was published in 2022. Journal: J Healthc Eng.

The outbreak of COVID-19 directly burdened the public health systems and even led to humanitarian disasters in several countries worldwide [4]. The immediate short-term impact of the epidemic was a burden on medical relief and supplies. Differences between the centralized and decentralized political systems of China and Western countries such as the United States led to differences in the allocation of emergency medical resources, specifically in terms of medical and material security. In terms of medical security, the nationwide concentration of medical resources to support Hubei province, the massive concentration of emergency medical resources in Wuhan city, and the completion of Mount Thor, Mount Vulcan, and a large number of module hospitals were the key to the success of China in preventing and controlling COVID-19. However, as the traditional global public health leader, the lack of centralized control in the United States led to a lack of medical treatment capability in the worst-hit areas [5]. Countries such as Italy also experienced panic for medical resources due to the lack of medical security capability [6]. Hence, it was evident that Western countries, represented by the United States, did not release accurate and timely information to the public and did not establish effective coordination within regions and countries. China devoted its national efforts to rapidly preventing the spread of the epidemic and strived to quickly enter a phase of regular epidemic prevention and control in emergency material support [3]. However, the intervention of politicians and special interest groups in the public policy decisions of the Trump administration led to a low rate of popular mask-wearing and a lack of effective coordination between regions and states [7]. The effects of epidemic prevention and control in China were outstanding across the world and praised by the World Health Organization [8]. Fluctuations from “emergency management” to “emergency governance” were realized based on the Chinese experience, such as the consultation and research mechanism, the military and local emergency rescue mechanism, and the flat emergency organization and command system. Therefore, China developed an innovative theory in national security, established a set of risk governance systems, and formed an institutional guarantee for the modernization of the national governance system and governance capability [9].

Possible research contributions were as follows: Previous studies explained the effectiveness and deficiencies of emergency response in epidemic prevention and control in China and proposed corresponding policy recommendations, but most of them were limited to theoretical studies; hence, the reliability of the findings needed further investigation [10–12]. Previous studies also lacked empirical findings on the effectiveness of epidemic response from the perspective of epidemic prevention and control and capital markets. As China is considered to be a model of epidemic response and governance among the current emergency response in the world [13], whether the deficiencies proposed in previous studies are weaknesses in emergency response needs in China are to be examined by empirical research methods. This paper examined the effectiveness and deficiencies of emergency management in the prevention and control in China, using empirical models. Therefore, it provided a theoretical basis for improving the emergency governance system with Chinese characteristics in major public health emergencies, ideas, and references for the improvement in emergency governance, and insights for countries around the world to contain the global spread of the epidemic.

The article "Analysis of the Government and Capital Market's Response to Normalized Epidemic Prevention and Control Based on the Development of Smart Health Care" was published in 2022. Journal: J Healthc Eng.

## 2. Literature Review

Compared with Western countries in terms of emergency response, Chinese government departments rapidly improved material security capability and deployed emergency resources to enhance medical security capability, improved the reserve and deployment of medical resources in each city, and centralized the admission and isolation of patients during the prevention and control of COVID-19 [14]. Studies related to emergency response mainly focused on the response of public health emergency itself and the economic consequences.

### 2.1. Public Health Emergency Response

Previous studies on the response of public health emergency itself found that the medical talent allocation, material and equipment security, environment policy support, and medical information system application were the important factors influencing the emergency medical treatment capability [15]. In terms of medical talent allocation, Padilla-Elías concluded that emergency talent was currently a major shortcoming of public hospitals in public health emergency response [16]. In material and equipment security analysis, Ahmed et al. constructed a decision-making model for major public health emergencies based on the spatial and temporal characteristics, key events, transmission dynamics, spatial distribution, infection scale, information characteristics, and medical resource dimensions [17]. Hu et al. established observation indicators that significantly promoted the clarification of prevention and control priorities, achieved early warning effects, clarified the reserve direction of emergency medical resources, and prevented the recurrence and spread of COVID-19 [18]. In terms of medical information system application, Asadzadeh et al. proposed the different effects and intrinsic mechanisms of direct and indirect applications of medical information systems on the quality of clinical treatment services and the quality of doctor-patient communication [19]. Based on macrogovernance, coordination management system, normalized guarantee mechanism, and medical security mechanism for major epidemics, Xiong et al. continued to improve the theoretical basis for major public health emergency response, such as the prevention system of public health emergencies, emergency response mechanism, social mobilization mechanism, financial investment, and international cooperation mechanism, so as to reform and improve the existing public health emergency governance system in China [20].

The article "Analysis of the Government and Capital Market's Response to Normalized Epidemic Prevention and Control Based on the Development of Smart Health Care" was published in 2022. Journal: J Healthc Eng.

Scholars also studied emergency response at the theoretical level. Gilson et al. analyzed the strategies of multiple actors in the prevention and control of major public health emergencies using the Grounded Theory [21]. Saeed et al. proposed opinions on the emergency response based on the space cooperation model [22]. Based on governance systems and institutions, Yin and Zhang evaluated the successes and deficiencies of the prevention and control of COVID-19 in China and proposed corresponding policy recommendations on the deficiencies, such as the lack of local government emergency response capability, delayed supply of emergency supplies, insufficient effective social mobilization, and weak public awareness of infectious epidemic prevention and control [23].

### 2.2. Economic Consequences of Emergency Response

Studies on the economic consequences of the emergency response generally found that COVID-19 had a significant impact on the economy. For example, Liu et al. found that the continued development of COVID-19 affected the economy of China in terms of lower output, reduced consumption, lower investment, restricted foreign trade, industrial development, and risks to financial institutions [24]. The economic development of China is in a critical stage, and it is vital to strive for sustained and stable economic development after COVID-19. At the macro level, He et al. investigated that the rapid spread of COVID-19 would lead to violent shocks in the global stock market and an effective mechanism to manage the impact of the epidemic on the world economy lacked worldwide. He proposed an emergency response mechanism and risk prevention strategies for macro governance in COVID-19 to control the negative impact of COVID-19 on the world economy [25]. At the microlevel, Mezghani et al. found that the crisis would reduce the investment willingness of listed companies, but the reduction was temporary [26]. Wang and Zhang studied the contribution of finance in socioeconomic resilience under the background of COVID-19 and proposed that financial policies had a significant impact and could significantly enhance socioeconomic resilience [27].

The article "Analysis of the Government and Capital Market's Response to Normalized Epidemic Prevention and Control Based on the Development of Smart Health Care" was published in 2022. Journal: J Healthc Eng.

### 2.3. Literature Evaluation

Studies related to the emergency governance of COVID-19 investigated mostly the effects and deficiencies of emergency governance, but most of them were stated in the stage of theoretical research. Hence, the reliability of the research findings needs further testing. However, China is considered as a model for response and governance in the prevention and control of COVID-19 in countries around the world. Further investigation with an empirical research approach is required on whether the deficiencies presented in the existing literature are weaknesses in the emergency response of China. Therefore, this paper examined the situation of COVID-19, public health emergency governance mechanism of China, and its emergency response effectiveness, using an empirical model.

Countries around the world are facing all types of natural risks, human-caused risks, and emerging risks, leading to a paradigm shift from emergency management to emergency governance in emergency response and helping to establish a governance system from emergency prevention to emergency governance. Sun et al. found that medical treatment was a key response to the emergency governance of major public health emergencies represented by COVID-19 [28]. Bonalumi et al. proposed that medical resources in each city were the fundamental guarantee of medical treatment, especially in fever clinics and material reserves [29, 30]. The Chinese experience showed that the danger of the virus and the speed of its transmission were often poorly understood by the public at the beginning of the outbreak due to its complexity, multiplicity, and severity. For example, Wu et al. found that emergency identification and control were the primary aspects of emergency response in major public health emergencies. The emergency response in China focused on identification, isolation, and treatment, in which the top priorities were the beds, human resources, and material reserves [31]. Sansa came to a similar conclusion, finding that the urban medical treatment capability determined by beds, human resources, and material reserves was an important factor affecting the effectiveness of the emergency response. He proposed that the shortage of medical resources forcing a large number of patients to be isolated at home was widely considered to be an important factor in the slower decline in patient numbers in countries such as the United States [14].

The article "Analysis of the Government and Capital Market's Response to Normalized Epidemic Prevention and Control Based on the Development of Smart Health Care" was published in 2022. Journal: J Healthc Eng.

Based on previous research and after reviewing the response of China to COVID-19, the rapid deployment of resources by various departments, the centralized treatment and isolation of patients, and the effective control of the source of infection were the key measures in achieving significant strategic results in the prevention and control of COVID-19. Particular attention was paid to the medical resources of the cities, especially to the fever clinics and the material reserves. If the aforementioned theoretical analysis “the urban medical treatment capability determined by beds, human resources, and material reserves is an important factor affecting the effectiveness of emergency response” was valid, China could actively strengthen the medical and material security mechanisms. Therefore, the following hypotheses were proposed:

  H1: The severity of the epidemic situation is negatively correlated with the effectiveness of the emergency response.
  H1a: The improved emergency response reverses to promote the medical security capability.
  H1b: The medical security capability reverses to promote the material security capability.
  Investors' sentiments and the real economy may indirectly have an impact on stock market price fluctuations. Sansa proposed that stock markets in all major affected countries and regions changed after COVID-19, and all financial markets in China and the United States (e.g., Shanghai Stock Exchange and New York Dow Jones) had a significant positive correlation with the confirmed cases of COVID-19 [32]. Al-Awadhi et al. investigated that the variables caused by the emergence of COVID-19, such as the daily increase in the total number of confirmed cases and the daily increase in the total number of deaths, had a significant correlation with the stock returns of all companies [33]. Liu et al. evaluated that investors, listed companies, financial institutions, and academic circle changed their perceptions of the effectiveness of the disposition of major public events that occurred and triggered high investor sentiments, based on the positive index for the pharmaceutical services, software, and other service sectors and the negative index for the transportation, accommodation, and food service sectors [34–36]. The capital market becomes a sentiment-like indicator of feedback to the emergency medical security mechanism. This paper argued that COVID-19 had a correlation with average stock market trading volume. It further tested the association between the effectiveness of governance on COVID-19 and the investor confidence so as to examine whether the emergency response brought pressure to the capital market.
  H2: Capital market shows a positive market response to regions where emergency medical security mechanisms are effective.

The article "Analysis of the Government and Capital Market's Response to Normalized Epidemic Prevention and Control Based on the Development of Smart Health Care" was published in 2022. Journal: J Healthc Eng.

## 3. Data and Methods

### 3.1. Sample and Data Resource

This paper selected the daily data of Chinese provinces from January 10, 2020, to June 22, 2021, and obtained 11421 observations after excluding missing data for the main variables. The continuous variables involved were winsorized by 1% up and down to eliminate the effect of extreme values. All data are taken from the China Stock Market & Accounting Research (CSMAR) Database.

### 3.2. Variable Selection

In this paper, the natural logarithm of the sum of “1” and the number of new cures for each province was chosen to measure the dependent variable “emergency response” (NCs); the natural logarithm of the sum of “1” and the number of new confirmed diagnoses for each province was chosen to reflect the explanatory variable “epidemic situation” (NCDs); the natural logarithm of the sum of “1” and the number of fever clinic for each province was chosen to investigate the mesomeric effect of the medical security mechanism in each province; the natural logarithm of the sum of “1” and the number of emergency material enterprises for each province was chosen to measure the moderator variable “material security mechanisms” (EME).Thus, the trading volume could directly reflect the amplitude of changes in their expectations. Under the tremendous pressure brought by the epidemic to the Chinese economy, the increase in stock trading volume reflects the optimistic expectations and high sentiments of investors in the capital market. Therefore, this article uses the natural logarithm of the sum of “1” and the average stock market trading volume to measure “investor sentiment” (EME). This model incorporated four indicators reflecting the economic strength of local governments as control variables, such as natural logarithm of GDP by province (GDP), provincial industrial enterprise average scale (Size), provincial industrial enterprise leverage (Lev), and provincial tax revenues (Tax), to control the impact of the unequal economic strength of each province on the effectiveness of the emergency response. The definitions of all variables are listed in Table 1.

### 3.3. Empirical Modeling

Based on related research, this paper examined “pandemic situation-emergency medical security mechanism-emergency response effect,” and the following models were constructed:

(1) $$\begin{array}{c} {\text{FC}}_{t}=\beta_{0}*\text{NCD}s_{t-1}+\beta_{1}*X_{t}+\lambda_{t}+\varepsilon_{t}, \end{array}$$

(2) $$\begin{array}{c} \text{NC}s_{t+1}=\beta_{0}*{\text{FC}}_{t}+\beta_{1}*X_{t}+\lambda_{t}+\varepsilon_{t}, \end{array}$$

(3) $$\begin{array}{c} \text{NC}s_{t+1}=\beta_{0}*\text{NCD}s_{t-1}+\beta_{1}*{\text{FC}}_{t}+\beta_{2}*X_{t}+\lambda_{t}+\varepsilon_{t}. \end{array}$$

In model (1), FC_t_ was the natural logarithm of the sum of “1” and the number of fever clinics in each province in period *t*, and NCDs_*t*−1_ was the natural logarithm of the sum of “1” and the number of new diagnoses in each province in period *t* − 1; this was the same in models (2) and (3).

The article "Analysis of the Government and Capital Market's Response to Normalized Epidemic Prevention and Control Based on the Development of Smart Health Care" was published in 2022. Journal: J Healthc Eng.

In model (2), NCs_*t*+1_ was the natural logarithm of the sum of “1” and the new cures number in each province in period_*t*+1_; the same was in model (3). *X*_*t*_ was a set of control variables, *λ*_*t*_ was a time-fixed effect, and *ε*_*t*_ was a residual term.

Tobit regression was performed for model (1), and OLS regression was performed for model (2) and model (3). When the epidemic institution was severe, each province strengthened the emergency medical security mechanism, and then *ß*_0_ in model (1) was expected to be significantly positive. When the emergency security mechanism produced positive effects, then *ß*_0_ in model (2) was expected to be significantly positive. When the provinces improved the epidemic institution through the emergency medical security mechanism, then *ß*_0_ in model (3) was expected to be significantly positive.

This section further tested the moderating effect of the material security mechanism by constructing model (4) to examine the valid boundaries of the aforementioned findings:

(4) $$\begin{array}{c} \text{NC}s_{t+1}=\beta_{0}*\text{NCD}s_{t-1}+\beta_{1}*\text{NCD}s_{t-1}*\text{EME}+\beta_{2}*\text{NCD}s_{t-1}*\text{EME}+\beta_{3}*X_{t}+\lambda_{t}+\varepsilon_{t}. \end{array}$$

OLS regression was performed for model (4). *ß*_1_ was expected to be significantly positive when good material security could strengthen the emergency response effect of the medical security mechanism under the background of COVID-19.

## 4. Empirical Results and Analysis

### 4.1. Descriptive Statistics

Table 2 reports the descriptive statistics for the main variables. In the 11,421 samples of Chinese provinces from January 10, 2020, to June 22, 2021, the Min, Quartile 1, Med, and Quartile 3 of the natural logarithm of the sum of “1” and the number of new confirmed diagnoses for each province were 0; the Max was 8.072. The data showed that most samples from each province in China during COVID-19 had no new confirmed diagnoses, with only a few samples having a high number of new confirmed cases. Despite the high number of new confirmed diagnoses in the early stage of COVID-19, it was contained timely and effectively, and the overall control was effective.

The article "Analysis of the Government and Capital Market's Response to Normalized Epidemic Prevention and Control Based on the Development of Smart Health Care" was published in 2022. Journal: J Healthc Eng.

The minimum value of EME was 0, the maximum value was 4.934, and the mean and median were 2.271 and 2.303, respectively. The standard deviation was 1.500, which represented some variation in material security mechanisms between samples. However, overall, the distribution was relatively even and the differences were not significant. The minimum value of Ajygs was 15.532, the maximum value was 18.078, and the mean and median values were 16.587 and 16.503, respectively, which represented some variation in the material security capability of provinces and municipalities. All other variables were within a reasonable range of values.

### 4.2. Regression Result Analysis

Table 3 shows the data for each variable and the relationship between them.

Column 1 shows the measurement relationship between the number of new confirmed diagnoses and the number of fever clinics in the province in period *t* − 1, which was significantly positively correlated at the 1% statistical level. The medical security mechanism (FC) was strengthened in each province and city with severity in the epidemic situation (NCDs).

Column 2 shows the measurement relationship between the number of fever clinics in period *t* and the number of new diagnoses in period *t* + 1, which was significantly positively correlated at the 1% statistical level. The emergency response effect (NCs) sharply improved with a strengthening of the medical security mechanism (FC) in each province and city.

Based on the results in columns 1 and 2, column 3 verified the mesomeric effect of the medical security mechanisms, which were significantly positively correlated at the 1% statistical level. The results showed that the medical security mechanism in each province and city was an effective mechanism for improving the emergency response under the background of COVID-19 in China.

Column 4 verified the moderating effect of the number of material security mechanisms (EME) in each province, which was significantly positive at the 1% statistical level. The results showed that the regression coefficient of NCDs ∗ EME was 0.206, indicating that effective material security could significantly enhance the emergency response effect of the medical security mechanism in COVID-19, which showed that the material security mechanism was an important supplementary mechanism to the medical security mechanism.

### 4.3. Examination of the Relationship between Epidemic Response Effects and Stock Market Volume

Models (5)–(7) were constructed as follows to examine the impact of the epidemic situation on investor sentiment and the mesomeric effect of emergency response:

(5) $$\begin{array}{c} {\text{Ajygs}}_{t}=\beta_{0}{\text{FC}}_{t}+\beta_{1}*X_{t}+\lambda_{t}+\varepsilon_{t}, \end{array}$$

(6) $$\begin{array}{c} {\text{Ajygs}}_{t}=\beta_{0}\text{NC}s_{t}+\beta_{1}*X_{t}+\lambda_{t}+\varepsilon_{t}, \end{array}$$

(7) $$\begin{array}{c} {\text{Ajygs}}_{t}=\beta_{0}\text{NC}s_{t}+\beta_{1}\text{NC}s_{t}*{\text{FC}}_{t}+\beta_{2}{\text{FC}}_{t}+\beta_{3}*X_{t}+\lambda_{t}+\varepsilon_{t}, \end{array}$$

where Ajygs_t_ is the natural logarithm of the sum of “1” and the average stock market trading volume of listed companies for each province.

The article "Analysis of the Government and Capital Market's Response to Normalized Epidemic Prevention and Control Based on the Development of Smart Health Care" was published in 2022. Journal: J Healthc Eng.

Tobit regression was performed for model (5) and model (7). When the investors of the capital market presented a more positive sentiment to firms in regions with better emergency medical treatment capability, *ß*_0_ in model (5) was expected to be significantly positive. When the investors of the capital market presented a more positive sentiment to firms in regions with better emergency effects, *ß*_0_ in model (6) was expected to be significantly positive. When the emergency medical treatment capability of the region was identified by the capital market through emergency response effects, which resulted in a corresponding market response, *ß*_0_ was expected to be significantly positive in model (7).

Table 4 shows the connection between the emergency response mechanism, the emergency response effect, and investor sentiments.

Column 1 showed the measurement relationship between the number of fever clinics (FC) and the investor sentiment (Ajygs) in each province, which proposed that the number of fever clinics in each province was significantly and positively correlated with investor sentiment at the 1% statistical level, indicating that the investors of the capital market showed a more positive sentiment to firms in regions with higher emergency medical treatment capability.

Column 2 showed the measurement relationship between the number of new cures (NCs) and investor sentiments (Ajygs) in each province, which proposed that the number of new diagnoses in each province was significantly and positively correlated with investor sentiments at the 1% statistical level, indicating that investors of capital markets showed a more positive sentiment to firms in regions with significant emergency effects.

Column 3 showed the mesomeric effect of the number of new cures (NCs) in each province, which proposed that the number of new diagnoses (NCs) in each province mediated between the number of fever clinics (FC) and investor sentiment (Ajygs) in each province, indicating that the investors of the capital market showed a positive sentiment when the emergency medical coverage mechanism was effective.

The article "Analysis of the Government and Capital Market's Response to Normalized Epidemic Prevention and Control Based on the Development of Smart Health Care" was published in 2022. Journal: J Healthc Eng.

## 5. Conclusion

Based on the findings, policy recommendations are proposed as follows:

1. Optimizing regional emergency material reserves and establishing an efficient emergency material governance system.
2. The current emergency governance system for public health emergencies in China is based on unified leadership, comprehensive coordination, categorized governance, hierarchical responsibility, and local governance, which helps optimize the emergency material security system and places high demands on emergency material governance. With the impetus of the material security mechanism, China has been making use of big data technology to significantly improve the efficiency of emergency material security and further optimize regional emergency material security. Therefore, establishing an efficient and linked emergency material governance system is an important element of improving public health emergency governance.
3. Improving the rationality of medical resource layout.
4. The 2018 Wuhan Health Care Development Brief indicates that per capita medical resources in Wuhan far exceeds the national average. However, the period of deterioration of the pandemic trend in Wuhan reflects the limitations of China's capacity for emergency expansion and regulation to some extent. It showed that the average daily number of newly diagnosed cases exceeded more than 1000, and the medical resources such as the number of fever clinics, the number of beds, and the number of medical personnel were severely inadequate. Therefore, it is necessary to take into account the rational layout of medical resources in each province and city and to maintain a certain capability in epidemic prevention and control.
5. Strengthening financial coordination and supervision mechanisms, thus maintaining the safety and stability of capital markets.
6. Although public health events such as COVID-19 will have a certain impact on the stock market and investor sentiments of China (Yang et al., 2020), the capital market could effectively identify the effects of the emergency security mechanism. When the emergency effect was better, the investors of the capital market showed stronger sentiments. Therefore, it is important to strengthen the financial coordination and supervision mechanism to maintain the safety and stability of the capital market.

## Figures and Tables

**Table 1:** Definitions of variables.

Variable name	Variable notation	Variable definition
Emergency response	NCs	Natural logarithm of the sum of “1” and the number of new cures for each province
Medical security mechanism	FC	Natural logarithm of the sum of “1” and the number of fever clinic for each province
Epidemic situation	NCDs	Natural logarithm of the sum of “1” and the number of new confirmed diagnoses for each province
Material security mechanisms	EME	Natural logarithm of the sum of “1” and the number of emergency material enterprises for each province
Investor sentiment	Ajygs	Natural logarithm of the sum of “1” and the average stock market trading volume of listed companies for each province
Provincial GDP	GDP	Natural logarithm of GDP by province
Provincial industrial enterprise average scale	Size	Natural logarithm of the average scale of industrial enterprises by province
Provincial industrial enterprise leverage	Lev	Total liabilities/total assets of industrial enterprises by province
Provincial tax revenues	Tax	Natural logarithm of the sum of “1” and tax revenues for each province

Data source: CSMAR database.

The article "Analysis of the Government and Capital Market's Response to Normalized Epidemic Prevention and Control Based on the Development of Smart Health Care" was published in 2022. Journal: J Healthc Eng.

**Table 2:** Descriptive statistics of main variables.

Variables	Sample size	Mean	Standard deviation	Minimum value	Quartile 1	Median	Quartile 3	Maximum value
NCs	11,421	0.382	0.893	0.000	0.000	0.000	0.000	8.072
FC	11,421	5.702	1.438	0.000	5.529	5.858	6.501	7.540
NCDs	11,421	0.328	0.771	0.000	0.000	0.000	0.000	3.989
EME	11,421	2.271	1.500	0.000	0.693	2.303	3.638	4.934
Ajygs	11,421	16.587	0.584	15.532	16.111	16.503	17.041	18.078
GDP	11,421	10.955	0.328	10.353	10.767	10.877	11.107	11.725
Size	11,421	10.337	0.879	8.036	9.796	10.535	10.764	11.833
Lev	11,421	0.579	0.058	0.502	0.530	0.565	0.609	0.738
Tax	11,421	16.752	0.852	14.502	16.354	16.799	17.095	18.427

**Table 3:** Empirical tests of the epidemic situation, emergency response mechanisms, and effectiveness of the response.

Variable	(1) FC	(2) NCs_*t*+1_	(3) NCs_*t*+1_	(4) NCs_*t*+1_
NCDs_*t*−1_	0.052^*∗∗∗*^ (3.31)		0.437^*∗∗∗*^ (20.84)	0.808^*∗∗∗*^ (27.66)
FCt		0.030^*∗∗∗*^ (6.37)	0.021^*∗∗∗*^ (4.70)	
NCDst − 1 ∗ EME			*x*	0.206^*∗∗∗*^ (12.01)
EME				−1.568^*∗∗∗*^ (−14.47)
Date	0.000 (0.88)	−0.004^*∗∗∗*^ (−30.16)	−0.002^*∗∗∗*^ (−23.16)	–0.008^*∗∗∗*^ (−24.42)
GDP	0.762^*∗∗∗*^ (14.92)	−0.137^*∗∗∗*^ (–4.59)	−0.095^*∗∗∗*^ (−3.56)	−1.135^*∗∗∗*^ (−8.46)
Size	−0.893^*∗∗∗*^ (−21.53)	0.171^*∗∗∗*^ (7.16)	0.132^*∗∗∗*^ (6.48)	1.151^*∗∗∗*^ (9.57)
Lev	−1.480^*∗∗∗*^ (−5.45)	−1.369^*∗∗∗*^ (−7.09)	−1.242^*∗∗∗*^ (−7.11)	−9.072^*∗∗∗*^ (−12.44)
Tax	1.524^*∗∗∗*^ (33.48)	−0.007 (−0.24)	−0.025 (−1.02)	−0.145 (−1.12)
Annual	Control	Control	Control	Control
Constant term	−20.813^*∗∗∗*^ (−6.67)	79.019^*∗∗∗*^ (28.32)	52.836^*∗∗∗*^ (22.65)	177.544^*∗∗∗*^ (24.63)
Sample size	11,397	11,397	11,373	11,373
Pseudo R2	0.1179			
R-squared		0.164	0.288	0.1520

Note: *t*-statistics in parentheses; ^*∗∗∗*^, ^*∗∗*^, and ^*∗*^ indicate significance at the 1%, 5%, and 10% levels, respectively.

**Table 4:** Regression results of the emergency response mechanism, the emergency response effect, and investor sentiments.

Variable	(1) Ajygs	(3) Ajygs	(5) Ajygs
FC	0.018^*∗∗∗*^ (4.05)		0.017^*∗∗∗*^ (3.95)
NCs		0.021^*∗∗∗*^ (2.77)	0.020^*∗∗∗*^ (2.63)
Date	−0.000 (−0.12)	0.000 (0.81)	0.000 (0.77)
GDP	−0.421^*∗∗∗*^ (−18.13)	−0.406^*∗∗∗*^ (−17.65)	−0.418^*∗∗∗*^ (−18.03)
Size	−0.228^*∗∗∗*^ (−11.76)	−0.246^*∗∗∗*^ (−12.96)	−0.230^*∗∗∗*^ (−11.84)
Lev	0.134 (1.05)	0.128 (1.00)	0.143 (1.12)
Tax	0.110^*∗∗∗*^ (4.99)	0.135^*∗∗∗*^ (6.48)	0.108^*∗∗∗*^ (4.90)
Annual	Control	Control	Control
Constant term (math.)	21.690^*∗∗∗*^ (15.87)	20.086^*∗∗∗*^ (13.93)	20.461^*∗∗∗*^ (14.17)
Sample size	10,891	10,891	10,891
Pseudo R2	0.0865	0.0861	0.0869

Note: *t*-statistics in parentheses; ^*∗∗∗*^, ^*∗∗*^, and ^*∗*^ indicate significant at 1%, 5%, and 10% levels, respectively.

The article "Analysis of the Government and Capital Market's Response to Normalized Epidemic Prevention and Control Based on the Development of Smart Health Care" was published in 2022. Journal: J Healthc Eng.

## Data Availability

The datasets used and/or analyzed during the current study are available from the corresponding author on reasonable request.
